The article "Paeonol Suppresses Proliferation and Motility of Non-Small-Cell Lung Cancer Cells by Disrupting STAT3/NF-κB Signaling" was retracted in 2026. Reason: concerns about the images.

# Paeonol Suppresses Proliferation and Motility of Non-Small-Cell Lung Cancer Cells by Disrupting STAT3/NF-κB Signaling

**DOI:** 10.3389/fphar.2020.572616

**Published:** 2020-11-12

**Authors:** Lei Zhang, Wen-Xu Chen, Ling-Li Li, Yu-Zhu Cao, Ya-Di Geng, Xiao-Jun Feng, Ai-Yun Wang, Zhao-Lin Chen, Yin Lu, Ai-Zong Shen

**Affiliations:** ^1^ Department of Pharmacy, the First Affiliated Hospital of USTC, Division of Life Sciences and Medicine, University of Science and Technology of China, Anhui Provincial Hospital, Hefei, China; ^2^ Department of Pharmacy, Anhui Provincial Hospital, Anhui Medical University, Hefei, China; ^3^ Department of Pharmaceutics, College of Pharmacy, Anhui University of Chinese Medicine, Hefei, China; ^4^ Jiangsu Key Laboratory for Pharmacology and Safety Evaluation of Chinese Materia Medica, School of Pharmacy, Nanjing University of Chinese Medicine, Nanjing, China

**Keywords:** Paeonol, Non-small-cell lung cancer, STAT3, NF-κB, Cell motility, Cell invasion

## Abstract

**Background:** Targeting inflammatory microenvironment is a promising anti-tumor strategy. Paeonol is a phenolic compound with effective anti-inflammatory and anti-tumor properties. However, the effects of paeonol on non-small cell carcinoma (NSCLC) have not been fully investigated. Here, we evaluated the effects of paeonol on proliferation and metastasis of NSCLC and elucidated the underlying mechanisms.

**Methods:** The effects of paeonol on inflammatory cytokines were determined by cell proliferation and ELISA assays. Assays of wound healing, single cell migration and perforation invasion were used to evaluate migration and invasion of NSCLC cells. Expression of marker proteins in epithelial-mesenchymal transition (EMT) and matrix metalloproteinase (MMP) family enzymes were detected by Western blot assays. Nude mouse A549 cells transplantation tumor model was used to study the anti-lung cancer effects of paeonol *in vivo*. TUNEL stanining were used to detect the apoptosis of tumor cells in A549 lung cancer mice, and Ki67 analysis was used to detect the proliferation of tumor cells in A549 lung cancer mice. Immunohistochemistry was used to detect the effects of paeonol on signaling molecules in tumor tissues.

**Results:** Paeonol inhibited A549 cancer cell migration and invasion *in vitro*. Paeonol inhibited secreaion of inflammatory cytokines in A549 cells, including tumor necrosis factor (TNF)-α, interleukin (IL)-6, IL-1β, and transforming growth factor (TGF)-β. Paeonol altered the expression of marker proteins involved in EMT and MMP family enzymes. In addition, paeonol inhibited the transcriptional activity of nuclear factor-κB (NF-κB) and phosphorylation of signal transducers and activators of transcription 3 (STAT3). Paeonol inhibited the growth of A549 cells transplanted tumors in nude mice.

The article "Paeonol Suppresses Proliferation and Motility of Non-Small-Cell Lung Cancer Cells by Disrupting STAT3/NF-κB Signaling" was retracted in 2026. Reason: concerns about the images.

**Conclusion:** Paeonol potently inhibited NSCLC cell growth, migration and invasion associated with disruption of STAT3 and NF-κB pathways, suggesting that it could be a promising anti-metastatic candidate for tumor chemotherapy.

## Introduction

Lung carcinogenesis has been recognized as one of the hallmarks of human cancer, and recently shows a strong connection with inflammation (Altorki et al., 2019; Mohrherr et al., 2020). Approximately 25% of human cancers occur as a result of chronic inflammation. Epidemiological studies have shown that anti-inflammatory agents (such as aspirin, dexamethasone and ruxolitinib) can be beneficial for reducing the prevalence and mortality of cancer (Bock et al., 2014; Diakos et al., 2014). There are many similarities in cellular behavior, signal transduction and gene expression shared by cancer and inflammation, and both processes involve enhanced cell motility that is controlled by growth factors, cytokines, and inflammatory signals in tumor microenvironment. The infiltrated inflammatory cells produce different cytokines and chemokines to promote tumor cell migration and invasion and contribute to inflammation-mediated metastasis (Wu and Zhou, 2010; Yi et al., 2017).

Understanding the mechanisms by which inflammation contributes to tumor metastasis will lead to innovative approach for treating cancer. Cytokines and immune mediators promote tumor cell survival and chemoresistance through autocrine and paracrine mechanisms. Inflammatory cells produce tumor necrosis factor (TNF)-α (King, 2015), transforming growth factor (TGF)-β (Feng et al., 2017), interleukin (IL)-6 (Wouters et al., 2014), and other pro-inflammatory factors, which activate NF‐κB/STAT3 pathways and induce epithelial-to-mesenchymal transition (EMT) as well as cancer metastasis (Narayan and Kumar, 2012; Gray et al., 2014). Numbers of cancer-related cytokines frequently precede and contribute to NSCLC development (Zhang J. et al., 2019). Moreover, these cancer-related cytokines can activate several signal pathways, such as NF-κB and JAK/STAT, which control cancer cell proliferation, survival, and chemosensitivity (Ivanenkov et al., 2011; Garbers et al., 2015). Many pharmacological interventions have been developed to target inflammatory mediators and immune-related signal pathways. However, only a few of those have been demonstrated to be efficacious in clinical trials (Shaikh et al., 2019). Agents attacking multiple inflammatory signaling pathways may effectively prevent the proliferation and metastasis of tumor cells. Given the co-activation of NF-κB and STAT3 (two dominant pathways in inflammation and tumorgenesis) (He and Karin, 2011; Fan et al., 2013), small molecule inhibitors targeting them or the upstream receptors merit investigation for combination therapy for NSCLC.

The article "Paeonol Suppresses Proliferation and Motility of Non-Small-Cell Lung Cancer Cells by Disrupting STAT3/NF-κB Signaling" was retracted in 2026. Reason: concerns about the images.

Paeonol (2-hydroxy-4-methoxyacetophenone) has been used as an anti-inflammatory agent (Lou et al., 2017; Zhang L. et al., 2019; Zong et al., 2018; Al-Taher et al., 2020), and also has inhibitory effects on a wide range of cancers including pancreatic, ovarian (Saahene et al., 2018; Gao et al., 2019; Cheng et al., 2020)*,etc.* Recent studies revealed that paeonol could enhance the efficacy of chemotherapeutics, reduce cyclooxygenase-2 (COX-2) and regulate EMT by increasing Human Runt-Related Transcription Factor 3 expression in different types of tumors (Cai et al., 2014; Whittle et al., 2015). However, the underlying mechanism has not been elucidated yet. Given that chronic inflammation mediates tumor development and metastasis, we investigated the anti-tumor and anti-metastatic effects of paeonol on A549 NSCLC cells under inflammatory stimulation. Here, we report that paeonol potently inhibited A549 cancer cell migration and invasion associated with disruption of STAT3 and NF-κB pathways, suggesting that it may be a promising anti-metastatic candidate for lung tumor chemotherapy.

## Materials and Methods

### Reagents and Antibodies

Paeonol (purity >98%, HPLC) was purchased from the Xuancheng Herbs Plant Industry and Trade Co., Ltd. (Xuancheng, China) and was dissolved in dimethyl sulfoxide (DMSO) for all experiments. IL-6 and TNF-α were from Sigma (St Louis, MO, USA) and diluted to indicated concentrations for experiments. The primary antibodies used in Western blot analyses against STAT3, p-STAT3, IκBα, p-IκBα, p-NF-κB, and NF-κB were purchased from Cell Signaling Technology (Danvers, MA, USA). The primary antibodies against MMP-2, MMP-9, Bax, and Bcl-2 were from Santa Cruz Biotechnology (Santa Cruz, CA, USA). The primary antibodies against E-cadherin and N-cadherin were purchased from Signalway Antibody (Baltimore, MD, USA). The primary antibody against GAPDH and the horseradish peroxidase-conjugated secondary antibodies were obtained from Bioworld (St. Louis Park, MN, USA).

### Cell Culture

The NSCLC cell lines A549, H1650, and H1975 (Chinese Academy of Science, Shanghai, China) were grown in RPMI-1640 medium (Invitrogen, Grand Island, NY, USA) supplemented with 10% fetal bovine serum (FBS; Sijiqing Biological Engineering Materials Co., Ltd., Hangzhou, China), 100 U/mL penicillin and 100 mg/ml streptomycin. Cell morphology was assessed using an inverted microscope with a Leica Qwin System (Leica, Germany).

The article "Paeonol Suppresses Proliferation and Motility of Non-Small-Cell Lung Cancer Cells by Disrupting STAT3/NF-κB Signaling" was retracted in 2026. Reason: concerns about the images.

### Measurements of Cytokines

The secreted cytokines (TNF-α, IL-6, IL-1β, and TGF-β) in culture supernatant of A549 cells treat with or without paeonol were tested using ELISA (BD Biosciences, San Jose, CA, USA) according to the protocols provided by the manufacturer. The absorbance was read at 450 nm, with reference wavelength at 570 nm using a 96-well plate spectrometer (SpectraMax 190; Molecular Devices, Sunnyvale, CA). Calculation of the concentrations of the cytokines was performed in a log-log linear regression according to the instructions in the protocols.

### Cell Proliferation Assay

A549 cells in logarithmic growth were seeded in 96-well plates (5×103 per well) and cultured in RPMI-1640 medium supplemented with 10% FBS for 24 h, and then treated with 0.5% DMSO or paeonol at indicated concentrations or time periods. After treatment, 3-(4,5-dimethylthiazol-2-yl)-5-(3-carboxymethoxyphenyl)-2-(4-sulfo-phenyl)-2H-tetrazolium (MTS; Sigma, St Louis, MO, USA) and phenazine methosulfate (Promega Corporation, Madison, WI, USA) were added, and the cells were further incubated for 3 h at 37°C. The spectrophotometric absorbance at 490 nm was measured by a SPECTRAmax^™^ microplate spectrophotometer (Molecular Devices, Sunnyvale, CA, USA).

### Wound Healing Assay

24-Well plates were coated with 5% collagen for 1.5 h at room temperature, washed three times with phosphate buffered saline (PBS), and blocked by 2% bovine serum albumin (BSA)/RPMI-1640 medium. A549 cells were seeded at 1 × 10^5^ cells per well. Once the cells had attached properly, FBS-deprived medium and mitomycin (4 *μ*g/ml, Sigma, St Louis, MO, USA) were added to the cells for 3 h. One linear wound was scraped in each well with a sterile pipette tip, and cells were washed with PBS to remove the unattached cells. Then FBS-deprived medium was added to each well, and TNF-α or IL-6 with or without paeonol was added. Images were taken at indicated time points after wound induction using an inverted microscope with a Leica Qwin System (Leica, Germany). The number of cells migrating per millimeter of scratch was counted.

### Colloidal Gold Single Cell Migration Assay

Six-Well plates were coated with the colloidal gold particles. Serum-starved A549 cells were trypsinized and resuspended at a density of 1 × 10^3^ cells/mL. Suspension of 2 ml was added to each well. After incubation for 2 h, cells were pretreated with or without paeonol (20 *μ*g/ml) for 2 h, followed by stimulation with IL-6 or TNF-α for 24 h. When cells migrated, they phagocytized gold particles, resulting in corresponding white tracks. The single migrating cell was visible as a black body. Images were taken using an inverted microscope with a Leica Qwin System (Leica, Germany). Cell motility was evaluated by measuring the areas free of the gold particles using ImageJ.

The article "Paeonol Suppresses Proliferation and Motility of Non-Small-Cell Lung Cancer Cells by Disrupting STAT3/NF-κB Signaling" was retracted in 2026. Reason: concerns about the images.

### Transwell Invasion Assay

Cell invasion was evaluated using an 8 *μ*m pore size Transwell system (Millipore, USA). Briefly, the collagen stock solution (5 mg/ml), stored in −20°C, was thawed and mixed with RPMI-1640 medium and 1 M NaOH at a ratio of 1.37:0.22:0.1 at 4°C. The mixture (70 ml) was added onto the upper chamber. Serum-starved A549 cells were resuspended at a density of 5 × 10^5^ cells/mL. Cell suspension of 200 μl with or without paeonol upon stimulation with IL-6 or TNF-α were carefully transferred on the surface of collagen in the upper chambers. The bottom chamber was loaded with 0.8 ml of RPMI 1640 medium with 10% FBS. After incubation for 6 h, the filters were removed, rinsed two times with PBS, fixed in 4% paraformaldehyde and stained with 0.1% crystal violet. Cells on the upper side of the filter were wiped off with cotton swabs. The invasive cells in five random fields (×400) were counted and images were taken using an inverted microscope with a Leica Qwin System (Leica, Germany).

### Flow Cytometric Analyses of Apoptosis

Apoptosis was determined by FITC labeled annexin-V/PI double staining and flow cytometry analysis. A549 cells were treated with paeonol at indicated concentrations for 24 h. An Annexin V-FITC apoptosis assay kit (Nanjing KeyGen Biotech Co., Ltd., Nanjing, China) was used according to the protocol. Only fluorescein-positive cells without PI staining were regarded as apoptotic cells and the percentages were determined by flow cytometry (FACSCalibur; Becton, Dickinson and Company, Franklin Lakes, NJ, USA). The data were analyzed using the software CELLQuest.

### Western Blot Analysis

Whole cell protein extracts were prepared from treated A549 cells. The protein levels were determined using a BCA assay kit (Pierce, USA). Proteins (50 μg/well) were separated by SDS-polyacrylamide gel, transferred to a PVDF membrane (Millipore, Burlington, MA, USA), blocked with 5% skim milk in Tris-buffered saline containing 0.1% Tween 20. Target proteins were detected by corresponding primary antibodies, and subsequently by horseradish peroxidase-conjugated secondary antibodies. Protein bands were visualized using chemiluminescence reagent (Millipore, Burlington, MA, USA). Equivalent loading was confirmed using an antibody against GAPDH. The levels of target protein bands were densitometrically determined using ImageJ. The variation in the density of bands was expressed as fold changes compared to the control in the blot after normalized to GAPDH.

The article "Paeonol Suppresses Proliferation and Motility of Non-Small-Cell Lung Cancer Cells by Disrupting STAT3/NF-κB Signaling" was retracted in 2026. Reason: concerns about the images.

### Nuclear Translocation Assay

Cells were seeded in six-well plates and grown overnight. Cells were pretreated with paeonol for 24 h before stimulated with 20 ng/ml IL-6 or TNF-α for 10 min. Treated cells were washed with cold PBS followed by fixation with cold acetone for 10 min at 4°C. Cells were permeabilized with 0.5% Triton X-100 (Sigma, St. Louis, MO, USA) for 10 min at room temperature, washed with PBS and blocked with 1% BSA for 1 h. Antibody was added and incubated overnight at 4°C. After washing with PBS for three times, goat anti-rabbit IgG-Tritc was added and incubated for 1 h at room temperature. Fluorescence cells were observed and photographed under a laser scanning confocal microscope (LEICA, Mannheim, Germany).

### Luciferase Assay

NF-κB transcriptional activity was measured by a NF-κB-responsive luciferase reporter assay. In brief, A549 cells were seeded in 96-well plates and reached 70% confluence overnight. Luciferase reporter vector containing NF-κB response element and Renilla luciferase reporter plasmid as control were transfected into A549 cells for 24 h using X-tremeGENE HP DNA transfection reagent (Roche). Cells were then incubated with various concentrations of paeonol (5, 10, 20 *μ*g/ml) for 24 h. Before the indicated time, cells were stimulated with 20 ng/ml TNF-α or vehicle control for another 30 min. Relative transcriptional activity of 20 *μ*l of lysate/well sample was determined using the Dual-Luciferase Assay System (Promega).

### Animal Experiments

The *in vivo* research protocols were approved by the Animal Ethics Committee of Anhui Medical University. Male nude mice (18–20 g) were purchased from Changzhou Cavens Experimental Animal Co., Ltd., and subcutaneously injected with A549 cells suspension (1 × 105 cells in 0.1 ml per mouse) into the right forelimb of 15 nude mice. The mice were randomly assigned to the following three groups: group 1, NS group, intraperitoneal injection of normal saline; group 2, paeonol group, intraperitoneal injection of paeonol (50 mg/kg/d); group 3, cisplatin group, intraperitoneal injection of cisplatin (1mg/kg/d). Feeding and observing tumor growth, all nude mice were sacrificed 14 days after injection of tumor cells. TUNEL staining, immunohistochemistry and HE staining were performed according to standard procedures. Representative images are shown.

### Statistical Analysis

Data were presented as mean ± SD, and results were analyzed using SPSS16.0 software. The significance of difference was determined by one-way ANOVA with the post-hoc Dunnett’s test. Values of *p* < 0.05 were considered to be statistically significant.

## Results

### Paeonol Inhibits Proliferation and Secretion of Inflammatory Cytokine in A549 Cells

We initially determined the effects of paeonol on the morphology of three lines of NSCLC cells. The results showed that paeonol at 80 *μ*g/ml significantly altered the morphology of the three cell lines, and at 40 *μ*g/ml also remarkably affect the morphology of A549 cells. Paeonol at 20 *μ*g/ml or lower concentrations did not evidently change the morphology of the three cell lines (Figure 1A). These observations indicated that paeonol could affect the growth of various NSCLS cells but they had different sensitivity to paeonol treatment. To confirm this, cell proliferation was determined using MTS assays. Paeonol inhibited the proliferation of A549, H1650 and H1975 cells in concentration- and time-dependent manners. Paeonol at concentrations of 5–20 *μ*g/ml did not significantly reduce the proliferation of the three cell lines, but at 40 and 80 *μ*g/ml considerably inhibited their proliferation (Figure 1B). Notably, the IC50 value of paeonol inhibition of A549 cell proliferation was the lowest among the three cell lines, suggesting that A549 cells were mostly sensitive to paeonol treatment. Therefore, A549 NSCLC cells were selected for subsequent experiments. We additionally observed that paeonol at concentrations of 10 and 20 μg/ml did not appaently induce apoptosis in A549 cells and influence the protein expression of Bax and Bcl‐2 (Supplementary Figures S1A–C). These results directed us to investigate whether paeonol affected some other aspects of NSCLC cell biology at relatively low concentrations. Then we used ELISA methods to determine the levels of inflammatory cytokines (TNF-α, IL-6, IL-1β and TGF-β) in the supernatants of paeonol-treated A549 cells. The results showed that paeonol at 10, 20 and 40 μg/ml significantly reduced the supernatant levels of TNF-α and IL-6, IL-1β and TGF-β, respectively (Figure 2). These data suggested that paeonol at relatively low concentrations inhibited the secretion of inflammatory cytokines from A549 cells.

The article "Paeonol Suppresses Proliferation and Motility of Non-Small-Cell Lung Cancer Cells by Disrupting STAT3/NF-κB Signaling" was retracted in 2026. Reason: concerns about the images.

**FIGURE 1:** Paeonol inhibits proliferation in NSCLC cells. A549, H1650, and H1975 cells were treated with paeonol at indicated concentrations for 12, 24 or 48 h. **(A)** Representative morphological images of cells. Original magnification ×400. **(B)** MTS assays for evaluating cell proliferation, n = 3 (independent experiments). Signficance: *p < 0.05 vs. control, **p < 0.01 vs. control, ***p < 0.001 vs. control.

**FIGURE 2:** Paeonol reduces secretion of inflammatory cytokines in A549 cells. A549 cells were treated with paeonol at indicated concentrations for 24 h. ELISA was used to determine the levels of TNF-α **(A)**, IL-6 **(B)**, IL-1β **(C)**, and TGF-β **(D)** in supernatants, n = 3 (independent experiments). Significance: *p < 0.05 vs. control, **p < 0.01 vs. control, ***p < 0.001 vs. control.

### Paeonol Inhibits Motility in A549 Cells Stimulated by TNF-α or IL-6

We next turned to examined whether paeonol at concentrations less than or equal to 20 *μ*g/ml could regulate migration and invasion of A549 cells in the presence of inflammatory cytokines TNF-α (20 ng/ml) or IL-6 (20 ng/ml). Wound healing assays showed that both TNF-α and IL-6 significantly increased A549 cell migration, whereas paeonol significantly inhibited the migration of A549 cells not only under normal conditions but also upon the stimulation of TNF-α and IL-6 (Figure 3A). Colloidal gold single cell migration assays were used to further demonstrate the paeonol effects on A549 cell migration. The results were consistent with the observations in wound healing assays, showing that paeonol has a more effective inhibitory effect on TNF-α-induced A549 cell migration (Figure 3B). Cell invasion was examined by transwell invasion assays showing that TNF-α or IL-6 significantly promoted A549 cell invasion, whereas these stimulatory effects were significantly abolished by paeonol (Figure 3C). Taken together, these results indicated that paeonol suppress motility of A549 cells under stimulation of TNF-α or IL-6.

**FIGURE 3:** Paeonol represses motility in A549 cells stimulated with TNF‐α or IL‐6. A549 cells were treated with paeonol at indicated concentrations and/or TNF-α (20 ng/ml) or IL‐6 (20 ng/ml) for 24 h. **(A)** Wound healing assays with quantitation. **(B)** Colloidal gold single cell migration assays with quantitation. **(C)** Transwell invasion assays with quantitation. Representative images are shown from three independent experiments (n = 3). Original magnification ×400. Significance: **p < 0.01 vs. control, ***p < 0.001 vs. control, #*p* < 0.05 versus TNF‐α or IL‐6, ##*p* < 0.01 versus TNF‐α or IL‐6, ###*p* < 0.001 versus TNF‐α or IL‐6.

### Paeonol Modulates EMT and MMPs in A549 Cells

We subsequently explored the molecular mechanisms responsible for paeonol inhibition of A549 cell motility. We examined the effects of paeonol on the expression of N-cadherin and E-cadherin, two marker proteins in EMT, showing that paeonol concentration-dependently downregulated N-cadherin expression, but upregulated E-cadherin expression in A549 cells upon TNF-α or IL-6 treatment (Figure 4), suggesting that paeonol could inhibit the EMT process in A549 cells. Furthermore, paeonol reduced the protein expression of MMP-2 and MMP-9 in the presence of inflammatory cytokines (Figure 4), indicating that paeonol could inhibit matrix degradation. Altogether, these results indicated that alterations of EMT-related proteins and MMPs were associated with paeonol suppression of A549 cell motility.

The article "Paeonol Suppresses Proliferation and Motility of Non-Small-Cell Lung Cancer Cells by Disrupting STAT3/NF-κB Signaling" was retracted in 2026. Reason: concerns about the images.

**FIGURE 4:** Paeonol inhibits EMT and modulates MMPs system in A549 cells stimulated with TNF-α or IL-6. A549 cells were treated with paeonol at indicated concentrations and/or TNF-α (20 ng/ml) or IL-6 (20 ng/ml) for 24 h **(A,B)** Western blot analyses of N-cadherin, E-cadherin, MMP-9 and MMP-2 with quantification. GAPDH was used as an invariant control for equal loading and representative blots were from three independent experiments (n = 3). Significance: *p < 0.05 vs. control, **p < 0.01 vs. control, ***p < 0.001 vs. control.

### Paeonol Interrupts STAT3 Signaling and Inhibits STAT3 Nuclear Translocation in A549 Cells Stimulated by IL-6

Since the phosphorylation of STAT3 can be elevated by IL-6, we examined the effects of paeonol on STAT3 signaling in A549 cells stimulated with IL-6. As expected, paeonol inhibited phosphorylation of STAT3 in a concentration dependent manner (Figure 5A), suggesting that paeonol could block STAT3 signal transduction. In addition, nuclear translocation is critically important for STAT3 to exert its biological consequences as a transcription factor. Therefore, we further investigated whether STAT3 nuclear translocation was affected by paeonol. Immunofluorescence assays showed that STAT3 was primarily located in cytoplasm in the control cells, suggesting the inactive state of STAT3 signaling (Figure 5B). Treatment with IL-6 led to considerably increased STAT3 in the nuclear, but paeonol reduced IL-6-induced STAT3 nuclear translocation (Figure 5B), indicating that the transcriptional activity of STAT3 signaling was suppressed by paeonol. Altogether, these data suggested that paeonol could block IL-6-activated STAT3 signal transduction in A549 cells.

**FIGURE 5:** Paeonol disrupts STAT3 signaling in A549 cells stimulated with IL-6. A549 cells were treated with paeonol at indicated concentrations and/or IL-6 (20 ng/ml) for 24 h. **(A)** Western blot analyses of p-STAT3 and total STAT3 with quantification. GAPDH was used as an invariant control for equal loading and representative blots were from three independent experiments (n = 3). Significance: ***p < 0.001 vs. control, #*p* < 0.05 vs. IL-6, ##*p* < 0.01 vs. IL-6. **(B)** Immunofluorescence double staining for determining STAT3 nuclear translocation. Original magnification ×400. Representative images are shown from triplicate experiments.

### Paeonol Interrupts NF-κB Signaling and Inhibits NF-κB Transcriptional Activity in A549 Cells Stimulated by TNF-α

NF-κB as a key player was involved in inflammation-induced tumor metastasis. Thus, we further determined whether paeonol affected NF-κB signaling upon the stimulation of cytokines in A549 cells. The results showed that after TNF-α treatment, the NF-κB signaling pathway was obviously activated, and p-IκBα, IκBα, p-NF-κB p65, p-NF-κB p65 were significantly upregulated. However, paeonol concentration-dependently inhibited p-IκBα, p-NF-κB p65, and NF-κB, but the total protein IκBα, which serves as an inhibitor of NF-κB, was not apparently influenced (Figure 6A), indicating that the TNF-α-induced NF-κB signaling was blocked by paeonol. Similar to STAT3, nuclear translocation is also required for NF-κB signal transduction. Our detection of the nuclear translocation of NF-κB in the presence of TNF-α and/or paeonol revealed that the enhanced NF-κB translocation into the nucleus was abolished by paeonol in a concentration-dependent manner (Figure 6B). In addition, dual luciferase assays demonstrated that paeonol inhibited the transcriptional activity induced by TNF-α (Figure 7). Collectively, these data suggested that paeonol suppressed NF-κB signaling at *transcriptional level, contributing to the complete* interruption of NF-κB pathway in A549 cells.

The article "Paeonol Suppresses Proliferation and Motility of Non-Small-Cell Lung Cancer Cells by Disrupting STAT3/NF-κB Signaling" was retracted in 2026. Reason: concerns about the images.

**FIGURE 6:** Paeonol disrupts NF-κB signaling in A549 cells stimulated with TNF-α. A549 cells were treated with paeonol at indicated concentrations and/or TNF-α (20 ng/ml) for 24 h. **(A)** Western blot analyses of IκBα, p-IκBα, NF‐κB p65 and p‐NF‐κB p65 with quantification. GAPDH was used as an invariant control for equal loading and representative blots were from three independent experiments (n = 3). Significance: ***p < 0.001 vs. control, #*p* < 0.05 vs. TNF-α, ## *p* < 0.01 vs. TNF-α, ### *p* < 0.001 vs. TNF-α. **(B)** Immunofluorescence double staining for determining NF‐κB (p65) nuclear translocation. Original magnification ×400. Representative images are shown from triplicate experiments.

**FIGURE 7:** Paeonol inhibits TNF‐α‐induced transcriptional activity of NF‐κB in A549 cells stimulated with TNF‐α. A549 cells were treated with paeonol at indicated concentrations and/or TNF‐α (20 ng/ml) for 24 h. Dual‐luciferase assays were used to determine the transcriptional activity of NF‐κB, n = 3 (independent experiments). ***p < 0.001 versus control, #*p* < 0.05 versus TNF‐α, ##*p* < 0.01 versus TNF‐α.

### Paeonol Exerts Anti-Tumor Effects in Nude Mice With A549 Cell Transplantation

A549 cells were implanted subcutaneously in the right forelimb underarm of nude mice to construct an *in vivo* lung cancer model. After tumor formation, mice were continuously injected with saline, paeonol or cisplatin intraperitoneally for 14 days. The results showed that in the model, both paeonol and cisplatin showed inhibitory effects on tumor growth, and compared with the control group, the tumor volume of treatment groups was significantly reduced (Figure 8A). There was no significant weight loss in the paeonol treatment group, while the mice of cisplatin group began to lose weight from the day 6 (Figure 8B). Examinations of the weight and size of isolated tumors showed that paeonol and cisplatin had inhibitory effects on A549 cell xenografts (Figures 8C,D). Moreover, TUNEL staining was used to detect the apoptosis of tumor cells in mice transplanted with A549 cells. The number of TUNEL positive cells in the paeonol and cisplatin groups was significantly increased (Figure 9A). Analyses of Ki67 also showed that the cell proliferation rate in paeonol group and the cisplatin group was reduced, indicating that paeonol and cisplatin had inhibitory effects on tumor proliferation *in vivo* (Figure 9B). We also observed that the expression of p-JAK and p-STAT3 in paeonol group was lower than that in NS group, which was consistent with the effects of paeonol on A549 cells *in vitro.* Importantly, paeonol exhibited no toxic effects on non-tumor organs or tissues (Supplementary Figure S2), suggesting a high safety of paeonol. Altogether, paeonol had significant anti-tumor effects in nude mice with A549 cell transplantation with high safety.

The article "Paeonol Suppresses Proliferation and Motility of Non-Small-Cell Lung Cancer Cells by Disrupting STAT3/NF-κB Signaling" was retracted in 2026. Reason: concerns about the images.

**FIGURE 8:** Paeonol exerts anti-tumor effects on A549 cells transplanted tumors in nude mice treated with paeonol or cisplatin. **(A)** Tumor growth curve of A549 cells. **(B)** Body weights. **(C)** Tumor weights. **(D)** Morphological image of the tumors. Significance: *p < 0.05 vs. NS, n = 5.

**FIGURE 9:** Paeonol inhibits tumor cell growth and reduces the activation of JAK/STAT3 signaling in tumor tissue of nude mice transplanted with A549 cells. **(A)** Representative images of TUNEL immunofluorescence with quantification. **(B)** Representative image of Ki67 immunohistochemistry with quantification. **(C,D)** Representative images of p-JAK and p-STAT3 immunohistochemistry with quantification. Signficance: *p < 0.05 vs. NS, n = 5.

## Discussion

NSCLC represents a highly malignant and particularly aggressive cancer, and has characteristics of early, widespread metastases and poor prognosis (Wang et al., 2020). NSCLC metastasis is the main cause of significant morbidity and mortality associated with surgical resection, involving tumor cell motility, intravasation, and circulation in the blood or lymph system (Sadowska et al., 2011). Cisplatin, a platinum agent, due to its affinity for DNA and other intracellular nucleophiles, has strong anti-tumor activity against a variety of malignant tumors including lung cancer (Trendowski et al., 2019). However, cisplatin can also cause a variety of off-target toxicity (ototoxicity, nephrotoxicity, bone marrow suppression, and neurotoxicity), which not only seriously affects the quality of life of patients, but also leads to lower doses or the choice of alternative therapies that ultimately affect the results (Trendowski, et al., 2019). There is currently no effective measure to successfully alleviate these symptoms. Cisplatin toxicity is related to patient symptoms and genetic factors. For example, the single nucleotide polymorphism in acylphosphatase 2 and Wolfram syndrome type 1 gene is related to hearing loss caused by cisplatin (Trendowski, et al., 2019). Aging increases the risk of platinum-induced nephrotoxicity by 43%, which may be due to more comorbidities in elderly patients (Duan et al., 2018). The risk of nephrotoxicity in elderly patients in Asian countries is much higher than that in European countries and North America (Duan, et al., 2018). In addition, the production of pro-inflammatory cytokines (including TNF-α and IL-6) and inflammatory responses are considered important factors for cisplatin to damage these organs (Ozkok and Edelstein, 2014; Vasaikar et al., 2018). In the current study, our results showed that paeonol and cisplatin significantly inhibited the lung cancer of A549 cells. Although cisplatin had better anti-tumor effects than paeonol, cisplatin at therapeutic dose caused obvious kidney toxicity and partial liver damage evidenced by the immunohistochemical analyses of various organs and tissues. Paeonol had no side effects on the structure of liver and kidney tissues, suggesting that paeonol could be significantly better than cisplatin in terms of adverse reaction, which may be due to the anti-inflammatory effects of paeonol (Zhang L. et al., 2019).

The article "Paeonol Suppresses Proliferation and Motility of Non-Small-Cell Lung Cancer Cells by Disrupting STAT3/NF-κB Signaling" was retracted in 2026. Reason: concerns about the images.

It has been increasingly recognized that tumor microenvironment plays an important role in carcinogenesis (Mendes et al., 2020). Inflammation often exists in tumor microenvironment and is induced by inflammatory mediators produced by the tumor, stroma, and infiltrating cells. These factors modulate tissue remodeling and angiogenesis and actively promote tumor cell migration and invasion through autocrine and paracrine mechanisms (Liu et al., 2018). Many inflammatory mediators in tumor microenvironment link inflammation to tumor progression. Studies have demonstrated that TNF-α and IL-1β are required for the initiation of chronic inflammation and their activation of NF-κB pathway is closely related to tumor development (Jing and Lee, 2014). IL-6 is a major factor involved in inflammation-associated cancer strongly stimulating the activation of JAK and STAT3, and plays an important role in the spread and invasion of tumor cells (Yoon et al., 2012; Xiang et al., 2014). IL-6 can also be synergistic with cytokines such as TGF-β to induce EMT and thereby to promote tumor proliferation, motility and invasion (Lopez-Bergami and Barbero, 2020). Our present study found that paeonol concentration-dependently reduced the secretion of inflammatory cytokines from A549 cells, especially TNF-α and IL-6. Moreover, paeonol inhibited A549 cells migration and invasion upon TNF-α or IL-6 treatment.

A growing number of studies have indicated that EMT and MMP enzymes are critically involved in the enhanced motility and invasion of tumor cells (Wu et al., 2019). The event of EMT characterized by loss of E-cadherin and upregulation of N-cadherin can promote the transformation of tumor cell phenotype, rending the acquisition of fibroblast-like characteristics and leading to decreased cell adhesion and increased motility (Li et al., 2019). On the other hand, tumor cells can obtain increased ability to degrade extracellular matrix components via production and secretion of MMPs especially MMP-2 and MMP-9. Therefore, it could be much easier for tumor cells to permeate basement membrane and achieve distant invasion and metastasis (Pai et al., 2020). In the present study, we found that paeonol concentration-dependently downregulated the expression of N-cadherin, MMP-2 and MMP-9 and upregulated the expression of E-cadherin in A549 cells stimulated by both TNF-α and IL-6, suggesting that paeonol was able to reverse the EMT process. It could be postulated that modulation of EMT and MMPs might contribute to paeonol suppression of A549 cell migration and invasion. However, whether EMT and MMPs in A549 cells are regulated by inflammatory pathways awaits further investigation.

JAK3/STAT3 signaling plays a dual role in tumor inflammation and immunity because it critically links many carcinogenic pathways to inflammatory pathways. Increasing evidence has shown that blockade of JAK3/STAT3 signaling not only inhibits the proliferation of tumor cells, but also reduces the inflammatory promotion in tumor microenvironment. Activation of STAT3 by IL-6 prevents cancer cell apoptosis and promotes malignant cell proliferation via upregulation of proliferative and anti-apoptotic factors (Vaish and Sanyal, 2011). In the current studies, we demonstrated that paeonol inhibited IL-6-induced cell migration and invasion, and further found that STAT3 phosphorylation and nuclear translocation were reduced by paeonol in IL-6-stimulated A549 cells. These data suggested that IL-6-induced activation of STAT3 could be blocked by paeonol, which affected A549 cell motility and invasion. NF-κB as a transcription factor is commonly upregulated in cancer cells and is implicated in the increased synthesis of inflammatory cytokines (Liu et al., 2020). NF-κB not only activates genes associated with cancer cell proliferation, invasion and metastasis, but also induces the expression of inflammatory cytokines and chemokines (e.g., IL-6 and COX-2) (Hirano et al., 2020). NF-κB can crosstalk with STAT3 at multiple levels, and is also a critical target molecule for anti-tumor therapy (Degoricija et al., 2014). The IκBα phosphorylation is a key step for activation of NF-κB signaling. In the present study, we showed that paeonol concentration-dependently inhibited the NF-κB p65 phosphorylation and the subsequent downstream signaling mediators such as IκB induced by TNF-α in A549 cells. Then we confirmed that paeonol inhibited TNF-α-induced NF-κB nuclear translocation and transcriptional activity. These findings suggested that paeonol blockade of TNF-α/NF-κB signaling might be related to repressing migration and invasion in A549 cells. Given the crosstalk between NF-κB and STAT3, whether the blockade of IL-6/STAT3 signaling was due to the feedback regulatory mechanisms needs to be verified in further study.

The article "Paeonol Suppresses Proliferation and Motility of Non-Small-Cell Lung Cancer Cells by Disrupting STAT3/NF-κB Signaling" was retracted in 2026. Reason: concerns about the images.

## Conclusion

Our present studies demonstrated that paeonol inhibited the migration and invasion of A549 cells stimulated with IL-6 or TNF-α, and reduced the secretion of inflammatory cytokines in A549 cells. These effects might be associated with the inhibition of EMT and regulation of MMPs system. Molecular evidence showed that the STAT3 and NF-κB pathways were disrupted by paeonol, contributing to the inhibition of motility and invasion (illustrated in Figure 10). Paeonol also exerted potent anti-tumor effects in nude mice with high safety. Our results provided novel insights into the anit-tumor properties of paeonol implicated in anti-tumor therapy against NSCLC.

**FIGURE 10:** Proposed mechanisms of paeonol inhibition of cell motility in NSCLC cells.

## Data Availability Statement

The raw data supporting the conclusions of this article will be made available by the authors, without undue reservation.

## Ethics Statement

The animal study was approved by the Animal Ethics Committee of Anhui Medical University.

## Author Contributions

All authors listed have made substantial, direct, and intellectual contribution to the work and approved it for publication.

## Conflict of Interest

The authors declare that the research was conducted in the absence of any commercial or financial relationships that could be construed as a potential conflict of interest.

## Abbreviations

**Abbreviations:** BSA, bovine serum albumin; DMSO, dimethylsulfoxide; EMT, epithelial-to-mesenchymal transition; FBS, fetal bovine serum; IL, interleukin; MMP, matrix metalloproteinase; MTS, 3-(4,5-dimethylthiazol-2-yl)-5-(3-carboxymethoxyphenyl)-2-(4-sulfo-phenyl)-2H-tetrazolium; NF-κB, nuclear factor-κB; NSCLC, Non-small-cell lung cancer; PBS, phosphate buffered saline; STAT3, signal transducers and activators of transcription 3; TGF-β, transforming growth factor-β; TNF-α, tumor necrosis factor-α
